The article "EEG-Based Epileptic Seizure Detection via Machine/Deep Learning Approaches: A Systematic Review" was retracted in 2023. Reasons: signs of a paper mill; compromised peer review; unreliable results or conclusions.

# EEG-Based Epileptic Seizure Detection via Machine/Deep Learning Approaches: A Systematic Review

**DOI:** 10.1155/2022/6486570

**Published:** 2022-06-17

**Authors:** Ijaz Ahmad, Xin Wang, Mingxing Zhu, Cheng Wang, Yao Pi, Javed Ali Khan, Siyab Khan, Oluwarotimi Williams Samuel, Shixiong Chen, Guanglin Li

**Affiliations:** ^1^CAS Key Laboratory of Human-Machine Intelligence-Synergy Systems, Shenzhen Institute of Advanced Technology, Chinese Academy of Sciences, Shenzhen, China; ^2^Shenzhen College of Advanced Technology, University of Chinese Academy of Sciences, Shenzhen, China; ^3^Guangdong-Hong Kong-Macao Joint Laboratory of Human-Machine Intelligence-Synergy Systems, Chinese Academy of Sciences, Shenzhen, China; ^4^School of Electronics and Information Engineering, Harbin Institute of Technology, Shenzhen, China; ^5^School of Biomedical Engineering, Sun Yat-Sen University, Guangzhou, China; ^6^Department of Software Engineering, University of Science and Technology, Bannu, Khyber Pakhtunkhwa, Pakistan; ^7^Institute of Computer Science and Information Technology, The University of Agriculture, Peshawar, Khyber Pakhtunkhwa, Pakistan

## Abstract

Epileptic seizure is one of the most chronic neurological diseases that instantaneously disrupts the lifestyle of affected individuals. Toward developing novel and efficient technology for epileptic seizure management, recent diagnostic approaches have focused on developing machine/deep learning model (ML/DL)-based electroencephalogram (EEG) methods. Importantly, EEG's noninvasiveness and ability to offer repeated patterns of epileptic-related electrophysiological information have motivated the development of varied ML/DL algorithms for epileptic seizure diagnosis in the recent years. However, EEG's low amplitude and nonstationary characteristics make it difficult for existing ML/DL models to achieve a consistent and satisfactory diagnosis outcome, especially in clinical settings, where environmental factors could hardly be avoided. Though several recent works have explored the use of EEG-based ML/DL methods and statistical feature for seizure diagnosis, it is unclear what the advantages and limitations of these works are, which might preclude the advancement of research and development in the field of epileptic seizure diagnosis and appropriate criteria for selecting ML/DL models and statistical feature extraction methods for EEG-based epileptic seizure diagnosis. Therefore, this paper attempts to bridge this research gap by conducting an extensive systematic review on the recent developments of EEG-based ML/DL technologies for epileptic seizure diagnosis. In the review, current development in seizure diagnosis, various statistical feature extraction methods, ML/DL models, their performances, limitations, and core challenges as applied in EEG-based epileptic seizure diagnosis were meticulously reviewed and compared. In addition, proper criteria for selecting appropriate and efficient feature extraction techniques and ML/DL models for epileptic seizure diagnosis were also discussed. Findings from this study will aid researchers in deciding the most efficient ML/DL models with optimal feature extraction methods to improve the performance of EEG-based epileptic seizure detection.

The article "EEG-Based Epileptic Seizure Detection via Machine/Deep Learning Approaches: A Systematic Review" was retracted in 2023. Reasons: signs of a paper mill; compromised peer review; unreliable results or conclusions.

## 1. Introduction

Epileptic seizure is a well-known chronic neurological and noncommunicable disease, occurring in 4% to 16% of organ recipients and affecting between 60–70 million people worldwide [1]. Epilepsy can be observed at any age, with a higher incidence in infants and the elderly. Every year, around three million people are affected by this disease [1–4]. An epileptic seizure is a sudden abnormality in the brain's electrical activities, manifesting as excessive discharges of neuronal networks in the cerebral cortex and affecting the whole body [2]. It should be noted that the prediction of a seizure is hard, and for some patients, there may be hundreds of seizures in only one day, which may cause irreversible damage to the brain. Therefore, the timely detection and treatment of epilepsy are of great significance to control the development of the disease and improve the life quality of the patients. The most common causes include the shortage of oxygen during childbirth, malformations of organs, and low blood pressure [3, 4]. EEG (Electroencephalogram) is a method that records the neural electrophysiological activity of the brain by applying several electrodes over the subject's head with some criteria. EEG with different waveforms reflects different frequencies. By comparing, clinicians can diagnose some diseases related to the neural system. Several studies about epilepsy monitoring have been carried out based on electroencephalography (EEG) [5, 6], magnetoencephalography (MEG) [6], positron emission tomography (PET) [7], single-photon emission computerized tomography (SPECT) [8], functional magnetic resonance imaging (fMRI) [5], electrocorticography (ECoG) [9], and functional near-infrared spectroscopy (fNIRS) [9]. Compared to other techniques used in epilepsy, EEG signal devices are portable and economical, with their recordings being time-domain, and they can be transformed into frequency domain. EEG signals are produced by ionic currents from the variations in voltage coming from the brain's neurons, which show the brain's electric activity and are widely used in epileptic seizure detection [10, 11]. As shown in Figure 1, neuro-experts have categorized seizures based on the symptoms into two major categories, partial and generalized [4, 12]. A partial seizure can be defined by its symptoms, mainly caused by the affecting on the cerebral hemisphere.

The article "EEG-Based Epileptic Seizure Detection via Machine/Deep Learning Approaches: A Systematic Review" was retracted in 2023. Reasons: signs of a paper mill; compromised peer review; unreliable results or conclusions.

Moreover, a partial seizure can also be divided into two main groups: simple-partial and complex-partial. In the simple-partial, the person looks conscious and can generally communicate, while in the complex-partial, the patients behave abnormally, get confused, and typically act by chewing and mumbling. A generalized seizure also has two main parts. Nonconclusive seizure is diagnosed by obvious motor signs, while conclusive seizures are difficult to diagnose for having no motor signs. The person can only stare and not make additional motions or moments [12, 13]. In the epileptic seizure detection task, the neurologists analyze and diagnose the information reflected from EEG signals, such as the waveform, frequency, and amplitude, since EEG signals in a seizure will manifest some special indications like spikes. However, realizing the efficient detection of epilepsy seizures is frequently a time-consuming and exhausting task with the high possibility of human error, relying on clinicians' visual inspection. To be more specific, the limitations of manual epilepsy diagnosis can be listed as follows:

1. It requires the physicians to have plenty of experience in clinical diagnosis and professional skills, making it more subjective and possible for misdiagnosis. Besides, different clinicians may draw an inconsistent conclusion over the same EEG signals based on their experience [4].
2. EEG signals are weak electrophysiological signals, which means they are easily interfered with by noises and have a sharp decrease in their signal-to-noise ratio (SNR). EEG signals submerged in noise might have some changes in their waveform and make it difficult to diagnose [12].
3. The amount of EEG signals used to make a diagnosis of epilepsy is large. In the clinical setting, the EEG signals are usually recorded synchronously with video signals to help diagnose using some behavior indications, which further increases the clinicians' workload. It takes clinicians at least 16 hours to go through the EEG signals of the patients and make the diagnosis [11]. In clinical setting, the interruption of reviewing EEG signals and the heavy work load tremendously affect the clinician's judgments on the signals, which may cause misdiagnosis [13].

Based on the aforementioned limitation, finding a technique to solve those problems is worthwhile and important. With artificial intelligence (AI) development, computer-based prediction techniques, including machine/deep learning classifiers, may alleviate these challenges. In recent years, machine/deep learning techniques have been widely used in the clinical diagnosis of diseases, especially in the application of epileptic seizures. These machine/deep learning techniques greatly free the clinicians from the heavy workload, significantly improve the diagnosis efficiency, and provide an objective and accurate diagnosis. Moreover, the number of studies in this area using machine/deep learning (ML/DL) keeps growing rapidly.

The article "EEG-Based Epileptic Seizure Detection via Machine/Deep Learning Approaches: A Systematic Review" was retracted in 2023. Reasons: signs of a paper mill; compromised peer review; unreliable results or conclusions.

The keywords “EEG,” “Epilepsy,” “Epileptic Seizures,” “Deep Learning,” and “Machine Learning” were exploited to search articles. The keywords were searched in several citation databases, including IEEE, PubMed, Elsevier, Springer, Wiley, and ArXiv. In addition, Google Scholar was also utilized for further search.  Figure 2 shows the number of articles that have been accepted into each citation database. It has been noticed that IEEE, Elsevier, and Springer citation databases included the most accepted articles.

Initially, 400 accepted research articles were found in search engines. After keywords and title searches in each citation database, 200 articles were found.

Furthermore, full-text searches were conducted manually to select the best-accepted articles for review, 150 best potential articles were presented for the comprehensive review, and 50 articles were excluded. The first excluded criterion was the non-English articles. While the second excluded criterion represents the articles without availability of the performance metrics (accuracy, pre, sens, and spec), as shown in Figure 3.

In this paper, the main contribution is divided into four parts and is discussed as follows:

1. We have accomplished a comprehensive review of the three key dimensions. Firstly, the analysis of the statistical features and extraction methods of EEG signals in epilepsy seizures were achieved. Secondly, a systematic review of machine/deep learning models was conducted, including their performance, limitations, and associated challenges in epilepsy seizure datasets. Thirdly, we investigated the performance achieved by machine/deep learning models based on the logical results during adequate detection.
2. Throughout the research, we have found that a random forest model is more effective and efficient than other classifiers based on the adequate detection, and the random forest model handles high dimensional of the dataset and retrieves sensible information.
3. For further analysis, we have selected the time-domain feature extraction method with 9-statistical features (standard deviation, kurtosis, skewness, energy, line length, entropy, mean, mode, and Hurst) because they help the machine/deep learning models to retrieve relevant knowledge and the best logical result (accuracy of 98–100%).
4. The comprehensive review will help the researchers identify and use the most efficient machine/deep learning models with statistical feature extraction methods to improve the research in epileptic seizure detection.

The article "EEG-Based Epileptic Seizure Detection via Machine/Deep Learning Approaches: A Systematic Review" was retracted in 2023. Reasons: signs of a paper mill; compromised peer review; unreliable results or conclusions.

The paper distributions are as follows: Section 2 shows a framework for seizure detection.  Section 3 contains a detailed review of significant features and extraction methods, machine/deep learning models and challenges in seizure detection.  Section 4 presents results and discussion.

## 2. Epilepsy Detection and Classification Process

The procedure for epilepsy seizure detection and classification is described as follows:

### 2.1. A Framework of Seizure Detection

We present a framework of seizure detection using an EEG seizure dataset in the given context. Four steps are needed to accomplish the seizure detection process, including data collection and preparation, feature extraction and selection, and machine/deep learning techniques to classify the seizure. The whole framework of epileptic seizure detection is given in Figure 4.

### 2.2. Data Collection

Firstly, one of the most important parts to achieve seizure detection is data collection. It can be obtained using an EEG monitoring device to collect the EEG signals of the brain. The EEG monitoring device locates the EEG cap on the scalp area presented in 10–20 international systems [14]. The monitoring device records the electrical signals from different electrodes or channels connected with wires to the scalp's surface with various voltage and spatial information [15]. Moreover, these noisy EEG signals have been carefully investigated and monitored by the neuro-expert and categorized into ‘seizure' and ‘non-seizure' states.

### 2.3. Data Transformation

Data transformation is a difficult step after data collection, which converts the raw EEG signal data into a table format of 2-D. However, this relevant information is not sufficient for analysis to identify seizures. Various features' selection and modalities are applied to give precise information about a seizure.

### 2.4. Dataset Preparation

After successfully transforming the dataset (data transformation process), the next step is the preprocessing data phase. It is a data mining technique that transforms raw data into a meaningful and understandable format, removing null values, data reduction, and data cleaning of EEG seizure datasets [16].

### 2.5. Publicly Available Datasets

Using a dataset is crucial for data scientists and experts as it permits them to evaluate their proposed model's performance. Publicly accessible datasets are very important because they offer a benchmark to analyze the results by comparing each dataset. There are many online existing epilepsy-related datasets, and most of the recent research prefers to use the mentioned datasets, which are further illustrated as follows:

The article "EEG-Based Epileptic Seizure Detection via Machine/Deep Learning Approaches: A Systematic Review" was retracted in 2023. Reasons: signs of a paper mill; compromised peer review; unreliable results or conclusions.

#### 2.5.1. CHB-MIT—EEG Dataset

This dataset is generated at Children's Hospital Boston and the Massachusetts Institute of Technology (CHB-MIT) [17, 18] and is publicly accessible on a PhysioNet server. The dataset contains 23 patients: 5 men aged between 3 and 22 years and 17 girls aged from 1.5 to 19 years. Each patient has numerous seizure and nonseizure recording files in European data format (.edf).

#### 2.5.2. Bonn University—EEG Dataset

This dataset is split into five files (A–E) and includes 100 single-channel recordings. Each file has a record of 23.6 s, while all the signals have equal 128 channels recorded using 10–20 international electrodes system [19].

#### 2.5.3. Kaggle—EEG Dataset

The EEG dataset is part of the American Epilepsy Society's epileptic seizures detection challenge. It includes intracranial EEG signals from five dogs and two people who had 48 seizures spanning 627 hours. The EEG signals of dogs were recorded using 16 implanted electrodes, which were sampled at 400 kHz. In comparison, the EEG signals of patients 1 and 2 were recorded using 15 deep electrodes and 24 subdural electrodes, sampled at 5 kHz [20].

#### 2.5.4. Fribourg—EEG Dataset

This EEG dataset contains invasive EEG signals from 21 patients with refractory focal epilepsy monitored at the University Hospital of Fribourg's epilepsy center before surgery. The signals were collected during presurgical epilepsy monitoring. The intracortical grid, strip, and depth electrodes were used to provide direct recording from the focal area, reduce artifacts, and achieve a higher signal-to-noise ratio (SNR) [21].

#### 2.5.5. Bern Barcelona—EEG Dataset

The Barcelona database was compiled by the Bern Hospital's brain department in Barcelona, including intracranial EEG recordings from individuals who have focal epilepsy. Subjects were followed for many days without the use of antiepileptic medications to evaluate whether they were having seizures or needed surgery. The signals were collected using intracortical electrodes from AD-Tech, with one additional reference electrode located between the PZ and FZ positions [22].

#### 2.5.6. Zenodo—EEG Dataset

This dataset has multichannel EEG recordings of 79 human neonates recorded at Helsinki University Hospital, with an average recording length of 74 minutes. Three experts documented 460 seizures, 39 neonates were found to have seizures, and 22 neonates were seizure-free [23].

The article "EEG-Based Epileptic Seizure Detection via Machine/Deep Learning Approaches: A Systematic Review" was retracted in 2023. Reasons: signs of a paper mill; compromised peer review; unreliable results or conclusions.

Table 1 contains a list of the additional information for each dataset.  Figure 5 shows the number of each dataset used in epileptic seizures detection based on ML/DL techniques.

### 2.6. Feature Extraction and Selection Techniques Applied in Epilepsy Seizure Detection

Feature extraction is considered a core component of any pattern recognition system [24]. It is mainly because the feature extraction process often adopts a mathematically driven algorithm that helps extract relevant information mostly from a raw dataset to better characterize the pattern of interest at any given point in time. In many cases, integrating a feature extraction component in a pattern recognition system often leads to a better performance in accurately distinguishing various patterns of interest and yielding such results faster than the direct usage of the raw data [24]. Thus, feature extraction is considered necessary in developing an efficiently intelligent system for epileptic seizure detection. In the feature extraction stage of such a system, various approaches have been applied to the raw EEG signals toward obtaining information that allows the proper analysis of the underlying phenomenon of interest. The different commonly adopted feature extraction methods for EEG signal characterization are shown in Figure 6. After the feature extraction process task is completed, the resulting signals become more accessible and would certainly become highly informative for classifying the inherent seizure [25]. As mentioned earlier, it should be noted that using ML algorithms directly on the raw data set may produce low accuracy or even inconsistent results and most certainly require a relatively longer time to complete the prediction task [26]. Therefore, it is necessary to adopt a feature extraction technique, and at the same time, choose the best technique since there are several kinds of features for characterizing physiological signals, and selecting efficient statistical features is required when facing a challenging task.

Fundamentally, there are two ways in which features are often extracted from the EEG signal of interest, namely handcrafted and automatic extraction. The handcrafted extraction features are multivariate [27] and univariate in both frequency and time domains. In contrast, automatic features include mean [28], kurtosis, skewness, entropy [28], Horthy parameters, statistical moments, and variance [29]. Meanwhile, the most commonly adopted feature that is widely implemented in EEG signal characterization includes time-domain (TD), time-frequency domain (TFD), frequency domain (FD), fourier transform (FT), discrete wavelet transform (DWT), and continuous wavelet transform (CWT)-based features [30]. Abbasi et al. introduced wavelet scalograms (WSs) feature extraction techniques with DL models to detect HI brain injury and got satisfactory results [31]. Logesparan et al. [32] used various statistical feature extraction methods on EEG datasets but concentrated on only two features, “relative power” and “line length,” which produced better performance in seizure detection. Amin et al. [33] introduced tritime domain approaches for features selection with statistical features, namely line length, frequency, and energy in epilepsy seizure detection. They used CHB-MIT and BONN datasets to test the detection accuracy and reached 93–99% by calculating F-score, sensitivity, and specificity.

The article "EEG-Based Epileptic Seizure Detection via Machine/Deep Learning Approaches: A Systematic Review" was retracted in 2023. Reasons: signs of a paper mill; compromised peer review; unreliable results or conclusions.

Besides, many researchers implemented a single feature in epileptic seizure detection [34–36]. For example, Guo et al. [37] tested a single feature “line length” with machine learning classifiers ANN to classify EEG signal recordings, and the accuracy was 95.6%. Koolan et al. [34] introduced “line length” as a feature to detect seizures with a specificity of 85% and a sensitivity of 84%. Some researchers used a single feature, “line length,” while others applied many convenient features. However, many researchers have utilized other statistical features, which resulted in lesser accuracy (%) and more computational time (sec).

After feature extraction, one of the essential tasks is choosing a collection of informative, small, and compact features that have improved discriminating power. These features serve as the basic blocks for tasks, such as detection, classification, and regression, in biomedical signal processing. They are also one of the most important stages in the data analysis process. Indeed, features are a novel way of representing data, and they may be binary, categorical, or continuous. For example, characteristics, such as the patient's age, health condition, family history, electrode location, or EEG signal descriptors may be considered (voltage, frequency amplitude, phase, etc.). Therefore, it is suggested that the polynomial-based methods are used before applying machine-learning models to derive low-dimensional features. Usually, polynomial features aim to create/add new input features based on the existing features. The “degree” of the polynomial is used to control the number of features added, e.g., a degree of 3 will add two new variables for each input variable.

Different polynomial-based methods are available and may be used to decrease computation time and make more effective use of computer resources, which helps them become more popular [44]. Various efficient linear and nonlinear dimensionality reduction methods for feature selection in EEG-based epileptic seizure detection are shown in Table 2.

The article "EEG-Based Epileptic Seizure Detection via Machine/Deep Learning Approaches: A Systematic Review" was retracted in 2023. Reasons: signs of a paper mill; compromised peer review; unreliable results or conclusions.

## 3. Comprehensive Review of Efficient ML/Deep Learning Classifiers

Various pieces of literature have introduced machine/deep learning models for epileptic seizure detection using EEG signals datasets [45, 46] with statistical features methods and nonlinear parameters. In machine/deep learning models [47–53], random forest classifier (nonblack-box) and support vector machine (SVM), k-nearest neighbor (K-NN), artificial neural networks (ANN), convolutional neural network (CNN), recurrent neural networks (RNN), and autoencoder (AE) (“black-box”) are considered for review because of their remarkable performances in seizure detection.

### 3.1. Black-Box Classifiers in Seizure Detection

#### 3.1.1. Convolutional Neural Network (2D-CNN)

CNN is a popular deep learning classifier to predict and diagnose medical diseases [54]. Initially, CNN was used for image classification [55]. However, recent 1D-CNN has been modified to two-dimensionalarchitectures, broadly used to apply epileptic seizures and to process the EEG signal.  Table 3 presents a review of recent works that adopted 2D-CNN models to predict an epileptic seizure.

1D-CNN architecture is also a suitable choice for processing brain activity signals. Because 1D-CNN architecture requires less number of parameters; therefore, its detection time is less than 2D-CNN architecture but have worst classifcation performance. Therefore, 1D-CNN and 2D-CNN are capable of the diagnosis of epileptic seizures.  Figure 7 shows the seizure detection accuracies of the various kinds of literature-implemented 2D-CNN models [66–68].

#### 3.1.2. Recurrent Neural Networks (RNNs)

The sequential datasets, including videos, texts, and signals, have some characteristics, such as great length and variable, which is hard for a simple deep learning model to process [69]. RNNs model is widely used to overcome these challenges. RNNs are competitive models for processing biomedical signal data and receiving satisfactory results. The following section reviews RNN models commonly used in epileptic seizure detection with their corresponding accuracies.

The LSTM model was introduced after the RNNs drawbacks, short-term memory, and vanishing gradient [70–72]. Various pieces of literature using LSTM in seizure detection are available. Golmohammadi et al. [70] presented a 2-layer LSTM model and SoftMax function to evaluate the data and achieved 90% accuracy. The research of [73] demonstrated a 3-layer LSTM architecture model for classification and got satisfactory results, while the literature of [74] evaluated two hybrid models, GRU and LSTM, with the activator function. One of the layers is fully connected with a sigmoid activator in this network. The studies in [71–74] used 10 different architectures of RNN with 31 layers and got the best accuracy (95%).  Table 4 and Figure 8 present a review of recent works that adopted LSTM-RNN models to predict an epileptic seizure.

The article "EEG-Based Epileptic Seizure Detection via Machine/Deep Learning Approaches: A Systematic Review" was retracted in 2023. Reasons: signs of a paper mill; compromised peer review; unreliable results or conclusions.

#### 3.1.3. CNN_RNN

It is competent to use two models for more accurate diagnosis and prediction of epileptic seizures, such as CNN-RNN architecture. The structure of RNN helps process sequential data (time-series processing). In the literature of [82], they applied various preprocessing schemes and used a modified CNN-LSTM with 13 layers along with the sigmoid activation function in their last layers with 91% accuracy. Roy et al. [83] introduced a hybrid architecture CNN-RNN to achieve the best results. Their first experimental works consist of 1-D with a 7-layer hybrid model of CNN-GRU, and the second work has 3-D and CNN-GRU hybrid architecture. An extended study by Ravi Prakash et al. [84] implemented four deep learning architectures, and the accuracy of these experiments achieved 90.60%.  Table 5 and Figure 9 presented hybrid architectures (CNN-RNN) applied in different literature on epileptic seizures and their corresponding accuracies.

#### 3.1.4. Autoencoders (AEs)

Autoencoder (AE) is an unsupervised machine learning model that presents different input parameters and works with the function (compression, decompression) coupled with a neural network [88, 89]. The pieces of literature [45, 46, 90, 91] used multilayer autoencoders (MAE) to hybridize EM-PCA methods to reduce the dimensions for classification. They also implemented a genetic algorithm (GA), and the experimental results indicated an accuracy of up to 92.78%. Sharathappriya et al. [92] used stacked denoising AE (SDAE), which consisted of three layers of architecture. Qiu et al. [93] also introduced denoising sparse AE (DSpAE) and reported 95% accuracy. The study in [94] consisted of automated EEG with a machine learning-based system. This system has several parts: the first part extracted linear predictive cepstral coefficients (LPCC) as signal features. After that, three paths were used for accurate detection. They proposed SpAE to extract the feature from EEG, and SVM was used for the classification. Sharma et al. [48] achieved average accuracy up to 93.92%.  Table 6 presented AE in seizure detection and performance metrics, and an illustration of the authors of various literature with their accuracies was shown in Figure 10.

The article "EEG-Based Epileptic Seizure Detection via Machine/Deep Learning Approaches: A Systematic Review" was retracted in 2023. Reasons: signs of a paper mill; compromised peer review; unreliable results or conclusions.

#### 3.1.5. Conventional ML (ANN, SVM, KNN)

Based on their significant performances, SVM, ANN, and KNN have also been applied in various domains [73, 104], especially in processing brain signal datasets. Various relevant works listed here on seizure detection used different classifiers. Most of the research articles preferred hybrid models. Dorai and Ponnambalam [105] proposed a hybrid model using SVM and KNN to classify these EEG epochs into seizure and nonseizure types. Birjandtalab et al. [106] implemented a Gaussian mixture model (GMM) to diagnose epileptic seizure detection. They achieved satisfactory results of accuracy and an F-measure of 85.1%. This experimental work addressed the class imbalance issue in the given dataset. A detailed review of SVM, ANN, and KNN in seizure detection is shown in Table 7. The literature of [119] recommended ANN classifiers on the EEG brain activity dataset with time-frequency domain features. The implemented classifiers accurately classify the signals into “nonseizure” and “seizure” with 95% accuracy. They used the EEG dataset class combination from A to E. The proposed study by Satapathy et al. [120] applied two models, SVM and neural networks (“black-box” approaches), to the EEG dataset for seizure detection. The outcomes of the given models indicated that the SVM model was more efficient based on the accuracy and time complexity (sec) compared to other networks. Hassan and Subasi [122] used genetic algorithms (GA), SVM, and particle swarm optimization (PSO) to detect a seizure. This approach achieved the best accuracy up to 92.38%. Shoeb and Guttag [115] implemented SVM classifiers and vector features on the CHB-MIT dataset to predict seizures, achieving 93.38% accuracy. Amin et al. [33] also used four classifiers, namely Naïve Bayes, KNN, MLP, and SVM, for classification with the DWT method and relative features. Their experimental result showed 92% accuracy. Raghu et al. [117] introduced the hybrid KNN-SVM model that was implemented on raw EEG data for accurate classification of epileptic seizure detection, and the experimental result indicated an accuracy of up to 90%. Zabihi et al. [121] used an SVM classifier for specific accurate detection to process the dataset with frequency-domain and time-domain features and achieved 93.78% sensitivity and 96.05% specificity.

Lahmiri and Shmuel [125] successfully used the Hurst exponent (HE) to classify the recorded EEG dataset into nonseizure and seizure with up to 97% accuracy. Further study by Lahmiri and Shmuel [125] used SVM to accurately classify seizures with 100% accuracy but less time complexity (sec). Table 7 and Figures 11–13 showed the authors' accuracy of the three models (SVM, ANN, and KNN) in various pieces of literature.

The article "EEG-Based Epileptic Seizure Detection via Machine/Deep Learning Approaches: A Systematic Review" was retracted in 2023. Reasons: signs of a paper mill; compromised peer review; unreliable results or conclusions.

### 3.2. Nonblack-Box Classifiers in Seizure Detection

The issue of “black-box” classifiers is that it cannot identify human interpretation and classification procedures [128]. Therefore, there is less chance to retrieve sensible knowledge. Because of the limitation of knowledge retrievals, the researchers focus on “nonblack-box classifiers, including random forest and decision trees approach. The literature of [104, 129–132] examined the decision forest and decision tree, and they reported that decision forest classifiers were more effective than implementing a decision tree for its overfitting issues. An algorithm extracts the rules from training data using a decision tree that generates either a limited or a single set of logic rules (for example, whenever C2 entropy value is less than 101.01, class value = seizure) and stops growing the tree by adding more records to the training dataset once the rule is accepted by the algorithm [127]. Besides, the decision forest grows multiple decision trees on the training data with higher accuracy and sensible logic rules. Chen et al. [133] applied a decision tree on the EEG dataset to successfully classify seizures and reported 98.62% accuracy. Decision forest classifiers in [32, 134, 135] were used as ensemble methods for seizure detection, providing remarkable accuracy and creating additional logic rules with decision trees using the training data [120]. Siddiqui and Islam [136, 137] used the hybrid approaches of systematic forest (SySF) and continuously excluding root node (CERN) without epoch reduction to diagnose seizure detection. Another study [116] implemented decision forests with 9 statistical features with the epoch concept. The training dataset was divided into subdatasets, such as (d, d1,…, dn), and the accuracy was tested on each epoch. The limitation of this literature was that a single patient's dataset had been taken. The dataset could be taken from many patients to achieve the best results. Overall, a systematical review of recent studies and their performance of RF were presented in Figure 14 and Table 8. Because of the nonblack nature and advantages (accuracy, logic rules) [36, 139, 141], several researchers implemented a random forest classifier to diagnose seizure detection. Donos et al. [139] introduced a decision forest classifier on statistical features (frequency and time domains) extracted from the EEG dataset and reported that the system presented sensitivity up to 93.8%. Hosseini et al. [141] used the RF with grid search optimization (RF-GSO) approach and achieved an accuracy of 96.7%.

## 4. Observed Challenges from Surveyed Literature

Based on the comprehensive survey of existing related literature reviewed, it was observed that the various challenges in diagnosing epileptic seizures could be summarized as follows:

- The first challenge is that large epileptic seizure datasets are currently not available publicly for extensive validation of the proposed machine learning/DL-based models for epilepsy detection and classification.
- Many datasets only include specified chunks of EEG signals, which is insufficient for real-world applications, where detection must be done from real-time signals.
- Because a large amount of dataset is required for the proper validation of a machine learning model for epileptic seizure detection and classification, plenty of efforts have been made to combine available EEG datasets for this purpose. However, it is still difficult to combine these datasets because they have different parameters and were acquired under relatively different sampling conditions [142].
- Because machine/deep learning models mostly require substantial computational resources for their implementation in practical settings, which are sometimes difficult to access, a piece of good knowledge about how to optimize the models' performance is necessary for realizing a practical epileptic seizure detection and classification system.
- For some researchers working in epileptic seizure detection and prediction, especially those in low to medium-income countries, accessing high-performance hardware resources to implement deep learning models is often a key challenge. Although Google has made powerful computing servers accessible (Google Colab platform and so on), there are still limitations regarding the amount of data transferred to such servers and the length of time it takes for the servers to execute the tasks.

The article "EEG-Based Epileptic Seizure Detection via Machine/Deep Learning Approaches: A Systematic Review" was retracted in 2023. Reasons: signs of a paper mill; compromised peer review; unreliable results or conclusions.

## 5. Discussion

In this study, we have investigated the use of different machine/deep learning-based algorithms for epileptic seizure detection. For instance, the algorithms considered include the conventional ML (ANN, SVM, and KNN), advanced DL (CNN/RNN/LSTM), and the random forest (RF)-based ML because of their remarkable performances in epileptic seizure detection, as reported in previous studies.

A summary of the investigation results reported in recent literature are as follows:

This systemic survey indicates that conventional ML algorithms (ANN, SVM, KNN) contribute well to the processing of brain datasets (CHB-MIT, BONN, Kaggle, Fribourg, and Bern Barcelona) for seizure detection [106–120]. However, each method has some pros and cons. For instance, SVM is found to be efficient for binary classification. It has better detection accuracy than ANN and KNN, however, it has high computation time complexity (sec), mainly compared to KNN and ANN. In contrast, KNN has low-performance evaluation metrics (precision, recall, and F1-score), including low detection complexity, however, they can handle high dimensional datasets [111, 118, 125]. While introducing a hybrid classification scheme that involves a combination of machine learning models (SVM-KNN or SVM-ANN), an increase in detection accuracy, precision, recall, and F1-score can be achieved compared to using a single ML model [33, 108, 118, 126]. Even though hybrid models could achieve better prediction accuracy than single models, they are more computationally efficient than their single model counterparts, further limiting their implementation in practical applications [104, 132]. Additionally, a major challenge with conventional ML algorithms is that it is difficult to understand the logical procedure followed to arrive at their prediction outcomes and is largely unexplainable for patterns and the logic rules hidden inside the models (the blackbox concept). Thus, they are not recommended for extracting useful information from datasets.

On the other hand, advanced ML/DL (CNN/RNN/LSTM) aid the automatic extraction of high-dimensional features, which may not be easily achieved with conventional ML schemes. For instance, the RNN model is normally faster than CNN and LSTM in execution time but has relatively lower accuracy, precision, and recall. In contrast, LSTM has time complexity issues using CHB-MIT and BONN and other datasets for seizure detection [72, 77, 80]. Besides, the hybrid models (a combination of two or more DL models) were found to perform better in accurately classifying seizures at the expense of more computation time. When considering time complexity, accuracy, precision, and recall issues with the conventional ML and advanced ML (DL) algorithms, decision tree-driven schemes, such as random forest classifiers, may be good. It is partly because of their ensemble nature and multiple logic rules [127]. They can achieve fairly good classification results as shown in the previous sections [134–142]. Decision tree-based models can handle a relatively large number of datasets and are less time-consuming and mostly yield high accuracy, precision, and recall.

From adopting the conventional ML models for epileptic seizure detection, feature extract constitutes an essential component of the entire scheme. Hence, it is important to select proper feature extraction methods for characterizing the EEG signals. Recent studies that investigated and analyzed a range of features had indicated that the time-domain feature extraction methods with 9-statistical features (standard deviation, kurtosis, skewness, energy, line length, entropy, mean, mode, and Hurst) would be appropriate for epileptic seizure detection [126]. It is because the mentioned features have been reported to achieve average accuracies in the range of 98–100% when used with ML/DL models for epileptic seizure classification based on EEG signals.

The article "EEG-Based Epileptic Seizure Detection via Machine/Deep Learning Approaches: A Systematic Review" was retracted in 2023. Reasons: signs of a paper mill; compromised peer review; unreliable results or conclusions.

Furthermore, it is significant to select a smaller subset of useful features by adopting a selection technique to reduce the model's complexity. It leads to the survey of various feature selection methods adopted mainly for dimensionality reduction. The investigation study showed that Kernel principal component analysis (KPCA) was a suitable nonlinear reduction technique for feature selection. KPCA offers the following major benefits over other feature selection methods:

1. Nonlinear data is successfully handled.
2. No nonlinear optimization is required.
3. KPCA calculations are very easy and are similar to conventional PCA calculations.
4. The number of PCs does not need to be set before modeling [143].

KPCA is a suitable encoding method for data with a nonlinear manifold structure. It is widely used in various datasets, including applied health data, sensor data, and facial pictures.

## 6. Conclusion

A comprehensive review of efficient machine/deep learning models and feature extraction and selection methods has been performed in this research. This study focused on the conventional ML (ANN/SVM/KNN), advanced ML/DL (CNN/RNN/LSTM), and tree-base ML (RF) because of their remarkable performance in the application of epileptic seizure detection. This paper concluded that decision forest classifiers are the most suitable, effective, and recommended for future research in epilepsy seizure detection. Its nonblack-box nature produces explainable logic rules, multiple sensible knowledge (adequate detection), high accuracy, low detection complexity, high precision, and recall, reveals relevant information (seizure localization), and can handle high volumes of datasets. At the same time, blackbox classifiers, such as conventional ML (ANN SVM KNN) and advanced ML/DL (CNN/RNN/LSTM), cannot create logic rules, including high detection accuracy but have high time complexity.

Furthermore, according to the literature review, as for the selection of appropriate features and feature extraction method, we selected the time-domain features extraction method and 9-statistical features (standard deviation, kurtosis, skewness, energy, line length, entropy, mean, mode, and Hurst) because these features provided higher accuracy (%). At the same time, Kernel principal component analysis (KPCA) is a suitable nonlinear polynomial-based method for feature selection. Future research will further study machine learning issues regarding epileptic seizure detection with suitable features.

The article "EEG-Based Epileptic Seizure Detection via Machine/Deep Learning Approaches: A Systematic Review" was retracted in 2023. Reasons: signs of a paper mill; compromised peer review; unreliable results or conclusions.

## Figures and Tables

**Figure 1:** The illustration of seizure types and their subtypes.

**Figure 2:** The proportions of accepted paper for the review using different citation database.

**Figure 3:** A framework of how the systematic review was conducted.

**Figure 4:** A block diagram of epileptic seizure detection using EEG signals and machine/deep learning techniques.

**Figure 5:** Represents various datasets in different studies for epilepsy seizure detection using ML/DL techniques.

**Figure 6:** Different commonly adopted feature extraction methods for EEG signal characterization.

**Figure 7:** Comparison of accuracies (%) versus authors introducing 2D-CNN models for seizure detection.

**Figure 8:** Comparison of accuracies (%) versus authors introducing LSTM-RNNs models for seizure detection.

**Figure 9:** Comparison of accuracies (%) versus authors introducing CNN-RNN models for seizure detection.

**Figure 10:** Comparative study of accuracy (%) versus authors introducing AE model for seizure detection.

**Figure 11:** Comparative study of accuracy (%) versus authors introducing the SVM model for seizure detection.

**Figure 12:** Comparative study of accuracy (%) versus authors introducing the ANN model for seizure detection.

**Figure 13:** Comparative study of accuracy (%) versus authors introducing the KNN model for seizure detection.

**Figure 14:** Comparative study of accuracy (%) versus authors introducing RF model for seizure detection.

**Table 1:** Presents full description of publicly available EEG dataset datasets for epilepsy seizure detection.

Dataset	Recording	No. of seizure	Sampling frequency	Times	No. of patients
CHB-MIT [18, 19]	Scalp EEG	163	256	844	22
Bonn [20]	Surface and IEEG	NA	173.61	39 m	10
Freiburg [22]	IEEG	87	256	708	21
Kaggle [21]	IEEG	48	400/5 KHz	627	5 dogs, 2 patients
Zenodo [23, 24]	Scalp EEG	460	256	74 m	79 neonatal
Bern Barcelona [22]	IEEG	3750	512	83m	5

**Table 2:** Efficient polynomial-based methods for the features selection of EEG epileptic seizure detection.

Feature selection methods	Description
[38] principal component analysis (PCA)	It was implemented to compress highly correlated features into a lower-dimensional subspace and use in various pattern recognition applications, including EEG signal classification
[39] T-distributed stochastic neighbor embedding (t-SNE)	Used to decrease the dimensionality of nonlinear data with a high-dimensionality of complexity to a lower-dimensional subspace. It is extensively utilized to present large amounts of high-dimensional biological data
[40] kernel principal component analysis (KPCA)	Used to handle the problem of nonlinear dimensionality reduction and useful for data compression using electroencephalogram (EEG) signals
[41] independent component analysis (ICA)	Process multivariate data representing the vast database samples as EEG signal is composed of various random signals
[42] locally linear embedding (LLE) [43] generalized discriminant analysis (GDA)	One of the most frequently utilized methods for extracting the nonlinear features uses the EEG signal. GDA is a highly effective method for extracting the nonlinear features of EEG signal data because generalized discriminants are calculated by mapping the training data in large dimensions of space using a kernel function

The article "EEG-Based Epileptic Seizure Detection via Machine/Deep Learning Approaches: A Systematic Review" was retracted in 2023. Reasons: signs of a paper mill; compromised peer review; unreliable results or conclusions.

**Table 3:** A review of recent research that applied the 2D-CNN model for seizure prediction with their corresponding accuracies and limitations.

Authors	Machine-learning approaches	Feature selection methods	Dataset	Performance metrics	Limitations	Accuracy (%)
Bizopoulos et al. [56]	SoftMax, standard networks	2D and 3D phase space presents the intrinsic mode and functions	BONN	Overall accuracy	Low detection accuracy	85.30
Antoniades et al. [57]	LR, 2D-CNN	Time-domain	BONN	Overall accuracy	—	87.50
Park et al. [58]	SoftMax, 2D-CNN	2D, 3D phase space presents the intrinsic mode and functions	CHB-MIT, SNUH-HYU data	Spec, sens, time difference	Low sens, spec	90.58
Sui et al. [55]	SoftMax, 2D-CNN	FT	Kaggle	Overall accuracy	High time complexity	91.18
Turk and Ozerdem [59]	Softmax, 2D-CNN	Frequency-time domain, CWT	Freiburg	Spec, sens, acc, F-measure	Low spec for multi-class	93.60
Faust et al. [60]	Softmax, 2D-CNN	Wavelet transformations (DWT)	Bern-Barcelona data	Energy, frequency	Low accuracy	94.50
Tian et al. [61]	MV-TSK-FS, 2D-CNN	FFT, WPD	CHB-MIT	Overall accuracy	-	95.33
Lecun et al. [62]	Res-CNN	Conventional feature extraction method	BONN	Overall acc	-	95.70
LeCun and Triesch [63]	Softmax, 2D-CNN	Feature extracts from CNN	Bern Barcelona	Overall accuracy	High detection time	95.90
San-Segundo et al. [64]	SoftMax, 2D-CNN	DWT	CHB-MIT	Class acc	High training time	96.10
Akut [65]	Sigmoid, 2D-CNN	FFT, WPD	Kaggle	Spec, sens	High training time	96.15

**Table 4:** A review of recent research that applied the LSTM-RNN model for seizure prediction with their corresponding accuracies.

Authors	Machine learning approaches	Feature selection methods	Dataset	Performance metrics	Limitations	Accuracy (%)
Yao et al. [75]	SoftMax, LSTM	Independent RNN	CHB-MIT	Sen, spec, Prec	Low sens, prec	88.80
Chen et al. [72]	SoftMax, LSTM	Wavelet transformations (DWT)	Zenodo	Pre, spec, class	Low prec	90.00
Chen et al. [72]	SoftMax, LSTM	Wavelet transformations (DWT)	BONN	Overall accuracy	High detection time	91.82
Hussein et al. [76]	SoftMax, LSTM	Time domain, time-frequency domain	Fribourg	Sen, spec	—	92.75
Jaafar and Mohammad [77]	SoftMax, LSTM	Independent RNN	Freiburg data	Overall accuracy	High training time	93.75
Talathi and Vartak [78]	RNN, GRU	RNNs	BONN	Class accuracy	High time complexity	94.00
Ahmed-Aristizabal [79]	SoftMax, LSTM	Computer-based analytical approaches	Mater advanced epilepsy Unit	Overall accuracy	—	95.00
Yao et al. [80]	SoftMax, LSTM	Independent RNN	Bern Barcelona	Sen, spec, Prec	High time complexity	96.00
Hussein [81]	SoftMax, LSTM	Fully connected (FC) RNN	Zenodo	Sen, spec	High training time	96.00

The article "EEG-Based Epileptic Seizure Detection via Machine/Deep Learning Approaches: A Systematic Review" was retracted in 2023. Reasons: signs of a paper mill; compromised peer review; unreliable results or conclusions.

**Table 5:** A review of recent research that applied the CNN-RNNs model for seizure prediction with their corresponding accuracies.

Authors	ML/DL approaches	Feature selection methods	Dataset	Performance metrics	Limitations	Accuracy (%)
Fang et al. [82]	ST-GRU ConvNets	Time-domain	CHB-MIT	Latency	Low accuracy	77.30
Ravi Prakash et al. [84]	Sigmoid, 1D-CNN-LSTM	Time-domain features	Fribourg	Sen, spec	Low sens, spec	83.05
Ravi Prakash et al. [84]	CNN-RNN	2D, 3D phase space presents the intrinsic mode and functions	MAEU data	Overall accuracy	—	90.22
Ahmedt Aristizabal et al. [85]	Sigmoid, 2D CNN-LSTM	Time domain features	TUH data	Overall accuracy	High detection time	92.50
Roy et al. [83]	Sigmoid, 2D CNN-LSTM	Time-frequency domain feature	Kaggle	Sen, spec	High training time	93.00
Liang et al. [86]	Softmax, 1D CNN-GRU	2D, 3D phase space presents the intrinsic mode and functions	Bern Barcelona	Overall accuracy	High time complexity	94.16
Choi et al. [87]	ID-CNN biGRU	Frequency domain	CHB-MIT	Sensitivity	High training time	94.40

**Table 6:** A review of recent research that applied AE in seizure detection with their corresponding accuracies.

Authors	Machine learning approaches	Feature selection methods	Dataset	Performance metrics	Limitations	Accuracy (%)
Gasparini et al. [95]	SoftMax, SAE	Time-frequency, CWT	Reggio Calabria data	Sen, spec	Low Sen, Spec, Acc	86.50
Singh and Malhotra. [96]	SoftMax, SAE	AE and SE	BONN	Sen, spec, acc	Low Sen, Spec, Acc	88.80
Yuan et al. [97]	SoftMax, SSpDAE	SAE, six features	Zenodo	ROC, PR, F-measure	—	90.64
Yuan et al. [97]	SoftMax, SpDAE	Time-frequency	CHB-MIT	F1-measure, Confusion Matrix	Low detection acc	90.82
Hosseini et al. [98]	SoftMax, SpAE	PCA	Zenodo	Pre sen, FPR FNR	High FNR	91.00
Karim et al. [99]	SoftMax, SAE	DWT	BONN	Confusion matrix	Low prec	91.00
Yuan et al. [100]	SoftMax, SAE	AE and SE	CHB-MIT	Pre, sen, F-measure	—	92.61
Sharathappriyaa et al. [92]	SoftMax, AE	HWPT, FD	Fribourg	Sen, spec	High time complexity	92.67
Karim et al. [101]	SoftMax, SpAE	AE and SE	Fribourg	Confusion Matrix	High detection time	93
Karim et al. [102]	SoftMax, DSAE	ESD function	Kaggle	Sen, spec	—	94
Wang et al. [103]	SoftMax, SSpDAE	AE and NSP	BONN	Sen, spec	Prec not mentioned	95

The article "EEG-Based Epileptic Seizure Detection via Machine/Deep Learning Approaches: A Systematic Review" was retracted in 2023. Reasons: signs of a paper mill; compromised peer review; unreliable results or conclusions.

**Table 7:** Recently applied ML (SVM, ANN, and KNN) for seizure detection with their corresponding performances.

Authors	Machine learning approaches	Feature selection methods	Dataset	Performance metrics	Limitations	Accuracy (%)
Logesparan et al. [107]	SVM, ANN	Line length feature	CHB-MIT	ROC	Low accuracy	52
Zeiler Fergus [108]	QDA, DT, KNN, SVM	Time-frequency	BONN	Sen, spec	Low sen, pres	85
Birjandtalab et al. [106]	ANN	Spectral power	CHB-MIT	F-measure	High detection high	86
Chen et al. [109]	SVM	DWT	BONN	Confusion Matrix	Low sen, pres	86.83
Parvez and Paul [110]	LS-SVM	IMF, DCT-DWT, DCT, SVD	Freiburg	Spec, sen, Acc	Low sen, pres for binary classification	91.36
Guo and DiPietro [111]	K-NN	Genetic programming	BONN	Class Acc	Low accuracy	93.50
Nicolaou and Georgiou [112]	SVM	Permutation entropy	CHB-MIT	Pre, Rec, F-measure	Low prec and accuracy	93.55
Ahmad et al. [113]	SVM	DWT	CHB-MIT	Avg	—	94.8
Zhang et al. [114]	ELM, SVM	AE and SE	BCI Lab	Class accuracy	High time complexity	95.58
Shoeb and Guttag [115]	SVM	Time-frequency	CHB- MIT	Sensitivity (sen)	—	96
Chen et al. [116]	Naïve Bayes, SVM	Energy, variance, entropy, RMS	CHB-MIT	Pre, Rec, F-measure	Low pre	96.55
Raghu et al. [117]	RF, KNN, adaboost	Time-frequency	Bern-Barcelona	Sen, pre, NPR, ROC	NFR not mentioned	97.6
Mursalin et al. [118]	KNN, SVM, RF	15-features	BONN	Acc, sen, spec	—	98
Sharma et al. [119]	LS-SVM	2D, 3D phases, the intrinsic mode, and functions	BONN	Overall Acc	—	98.60
Amin et al. [33]	Naïve bayes, SVM, KNN, MLP	Energy	EPILEPSY	Class Acc	—	98.75
Satapathy et al. [120]	Neural network, SVM	CWT, DWT	BONN	Overall Acc	High detection time	99.1
Zabihi et al. [121]	SVM	Time-frequency	CHB-MIT	Sen, spec	High time complexity	99.32
Hassan and Subasi [122]	SVM	DWT	BONN	Class Acc	—	99.38
Fasil and Rajesh. [123]	SVM	Energy	BONN, Barcelona	Class Acc	—	99.5
Chen et al. [116]	LS-SVM	Entropies types	BONN	Spec, Acc, sen	—	99.58
Selvakumari et al. [124]	LS-SVM	DWT, FFT	Class Acc	BONN	High time complexity	100
Lahmiri and Shumel [125]	KNN and GHE		BONN	Class Acc	—	100
Kumar et al. [126]	DWT based approximate entropy ANN, SVM	DWT based approximate entropy	CHB-MIT	Overall Acc	High time complexity	100
Tzallas et al. [127]	ANN	Time-frequency features	BONN	Pre, Rec, F-measure	—	100

**Table 8:** A review of recent research applied random forest in seizure detection with their corresponding accuracies.

Authors	Machine learning approaches	Feature selection methods	Dataset	Performance metrics	Limitations	Accuracy (%)
Birjandtalab et al. [138]	Random forest-KNN	Spectral power	CHB-MIT	Sen, F-measure, prec,	Low sens, spec	80.87
Donos et al. [139]	Random forest	Time, frequency	EPILEPSY	Sensitivity	Spec not mentioned	93.8
Siddiqui et al. [140]	Random forest, boosting, decision forest	Nine statistical features	Bern Barcelona	Pre, Rec, F-measure	High time complexity	96.67
Wang et al. [137]	Random forest classifiers	Std, dev, energy, energy,STFT, mean	BONN	Class Acc	Low sens, spec for multi-class	96.7
Lee and Kim [35]	Random forest, SVM	Frequency, 10-time	UCI	ROC-AUC	—	98
Sharma et al. [119]	Random forest	IMF	Kaggle	Sen, spec, Acc	Sen, spec not mentioned	98.4
Mursalin et al. [118]	Random forest	DWT, entropy	Fribourg	Class Acc	—	98.45
Mursalin et al. [118]	Random forest	DWT, entropy	Zenodo	Class Acc	Sen, Spec not mentioned	98.45
Alickovic et al. [46]	ANN, random forest, SVM, KNN	Power, mean, kurtosis, absolute mean std dev, skewness	CHB-MIT	Sen, spec, Acc	Time complexity	100
Wang et al. [137]	Forest CERN	9-statistical features	BONN, CHB-MIT	Class Acc	—	100
Hosseini et al. [141]	Random forest classifiers	L1-penalized robust regression	BONN, CHB-MIT	Class Acc	—	100
